# A Rare Case of Solitary Schwannoma of Submandibular Gland

**DOI:** 10.7759/cureus.21373

**Published:** 2022-01-18

**Authors:** Sultan O Gohal, Saud S Alradadi, Abdullah A Althomali, Abdulrahman A Alshehri, Razan A Zabarmawi, Abdullah J Taha, Sommaya A Ajabnoor, Haya A Al Azmi, Atheer I Alqubaysi, Mohammed A Alshamrani, Nasser F Almutair, Ibrahim M Alotaibi, Saad A Alotaibi, Ahmed M Abdullah, Faisal Al-Hawaj

**Affiliations:** 1 College of Medicine, Batterjee Medical College, Jeddah, SAU; 2 Dentistry, Vision Colleges, Riyadh, SAU; 3 College of Medicine, Taif University, Taif, SAU; 4 Medicine, King Saud bin Abdulaziz University for Health Sciences, Riyadh, SAU; 5 Medicine, Ibn Sina National College for Medical Studies, Jeddah, SAU; 6 Medicine, Dar Al Uloom University, Riyadh, SAU; 7 Medicine, King Khalid University, Abha, SAU; 8 Medicine, King Saud University, Riyadh, SAU; 9 Medicine, Shaqra University, Shaqra, SAU; 10 College of Medicine, Imam Abdulrahman Bin Faisal University, Dammam, SAU

**Keywords:** case report, neck swelling, schwannoma, submandibular region, swelling

## Abstract

Tumors of the salivary gland constitute a heterogeneous group of variable histological and biological behaviors. Patients with salivary gland tumors typically present with painless swelling. However, several neoplastic and non-neoplastic pathologies can result in salivary gland enlargement. We report the case of a 35-year-old woman complaining of a left neck swelling for 3 months duration. She had no relevant past medical or surgical history. On examination, there was a left submandibular swelling that was firm in consistency, non-tender, non-pulsatile, relatively mobile, and was not tethered to the underlying structures. Otherwise, examination of the head and neck was unremarkable. A CT scan of the neck revealed a well-defined hypodense lesion in the left submandibular region with foci of calcification along with multiple enlarged lymph nodes. After surgical exploration, the submandibular gland region, a mass lesion was found arising from the submandibular gland. Histopathological examination revealed the diagnosis of schwannoma. Salivary gland schwannoma is a very rare form of neurogenic tumor. Surgical resection is the treatment of choice; however, neural deficits are important and common postoperative complications.

## Introduction

Tumors of the salivary gland constitute a heterogeneous group of variable histological and biological behavior. Such tumors are rare and account for only 6% of all head and neck malignancies. By far, the parotid gland is the most common site for salivary gland tumors [1,2]. However, only 25% of parotid gland lesions are malignant. In contrast, 50% of submandibular gland tumors are malignant. The most prevalent type of salivary gland tumor is a pleomorphic adenoma, while the most prevalent malignant type is mucoepidermoid carcinoma and adenoid cystic carcinoma. Patients with salivary gland tumors typically present with painless swelling [1]. However, several neoplastic and non-neoplastic pathologies can result in salivary gland enlargement. These include branchial cleft cysts, salivary gland stones, Sjogren syndrome, salivary cysts, and benign and malignant tumors [2]. Here, we report the case of a submandibular schwannoma, a rare tumor involving salivary glands.

## Case presentation

A 35-year-old woman presented to our family medicine clinic complaining of a left neck swelling. She noticed the swelling 3 months ago. It had been increasing in size gradually. However, it was not causing any symptoms and was completely asymptomatic. There was no history of overlying skin changes, ulceration, or discharge. She did not notice any other swelling. The patient reported no history of anorexia, weight change, or night sweats. No history of preceding upper respiratory tract infection. She had no relevant past medical or surgical history. She was a heavy smoker with 25 pack-years smoking history. She worked as an accountant. Her family history was significant for breast cancer.

On examination, there was a left submandibular swelling that was firm in consistency, non-tender, non-pulsatile, relatively mobile, and was not tethered to the underlying structures. Otherwise, examination of the head and neck was unremarkable. There was no regional lymphadenopathy. All cranial nerves were intact. Laboratory findings showed hemoglobin of 14.1 g/dL, leukocytes count of 8400/μL, platelets count of 384,000/μL. Further, the C-reactive protein (4.2 mg/dL) and erythrocyte sedimentation rate (11 mm/hour) were within the normal limits.

The patient underwent a neck ultrasound examination. It showed diffuse enlargement of the left submandibular gland that displayed a heterogeneous echogenicity and had a well-defined margin. No increased color blood flow was noted. Subsequently, a CT scan of the neck revealed a well-defined hypodense lesion in the left submandibular region with foci of calcification along with multiple enlarged lymph nodes (Figure 1). The clinical and radiological findings raised the possibility of submandibular salivary gland tumors, such as pleomorphic adenoma.

**Figure 1:** Axial (A), coronal (B), and sagittal (C) CT images of the neck showing a submandibular mass lesion (arrows) with foci of calcification CT: computed tomography

The patient was planned for surgical resection of this tumor under general anesthesia and no preoperative biopsy was taken. After exploration, the submandibular gland region, a mass lesion was found arising from the submandibular gland. The mass was successfully excised (Figure 2). The incision was closed and the patient recovered uneventfully. Histopathological examination showed elongated and wavy cells interspersed with collagenous fibers and it also revealed nuclear palisading and Antoni cells. Such findings represent the diagnosis of schwannoma (Figure 3). The patient was discharged after 3 days of hospitalization. She was followed up for 1 year and had no signs to suggest recurrence.

**Figure 2:** Gross pathology of the resected tumor

**Figure 3:** Histopathological image shows elongated and wavy cells interspersed with collagenous fibers in keeping with schwannoma

## Discussion

We report the case of a schwannoma involving the left submandibular region. Schwannoma is a common benign tumor arising from the Schwann cells [3]. However, schwannoma involving the salivary gland is very rare [4]. Such tumor may be seen at any age, but it is reported to be more prevalent among women. The first case of schwannoma of salivary glands was reported by Ellis [5] in 1991. Schwannoma may occur as a solitary lesion or as multiple lesions that could be associated with neurofibromatosis type 1. Malignant transformation of schwannoma is exceedingly rare [3].

Salivary gland schwannoma classically presents with a slow-growing painless mass. Pain due to the salivary gland schwannoma is considered very unusual [3]. The diagnosis of salivary gland schwannoma is made postoperatively in the vast majority of cases. MRI is the diagnostic investigation of choice to diagnose schwannoma and delineate its extent. It demonstrates a T1 signal intensity similar to that of skeletal muscles with a T2 signal intensity higher to muscles [6]. In the present case, the patient underwent a CT scan and the surgical decision was planned in a multidisciplinary meeting.

Schwannoma is considered resistant to radiotherapy making the surgical intervention necessary for optimal management. However, neural damages after surgical resection of salivary gland schwannoma are very common and are seen in more than 50% of cases. In the present case, however, the patient did not experience any neurological deficit after the surgical management [6]. The involved nerve was not identified in our case. Recurrence is very unusual in salivary gland schwannoma and the majority of case series reported no recurrence or malignant transformation of the lesion [7].

## Conclusions

Salivary gland schwannoma is a very rare form of neurogenic tumor. The clinical and radiological features of salivary gland schwannoma are usually non-specific. Hence, the diagnosis is often made postoperatively. Surgical resection is the treatment of choice; however, neural deficits are important and common postoperative complications. Despite its rarity, schwannoma should be remembered in the differential diagnosis of submandibular gland swelling.
